RETRACTED

# Immunosuppressant MPA Modulates Tight Junction through Epigenetic Activation of MLCK/MLC-2 Pathway via p38MAPK

**DOI:** 10.3389/fphys.2015.00381

**Published:** 2015-12-22

**Authors:** Niamat Khan, D. V. Krishna Pantakani, Lutz Binder, Muhammad Qasim, Abdul R. Asif

**Affiliations:** ^1^Proteomics Group, Institute for Clinical Chemistry/UMG-Laboratories, University Medical CentreGoettingen, Germany; ^2^Department of Biotechnology and Genetic Engineering, Kohat University of Science and TechnologyKohat, Pakistan; ^3^Department of Microbiology, Kohat University of Science and TechnologyKohat, Pakistan

**Keywords:** tight junction, permeability, MPA, epigenetic, promoter activity

## Abstract

**Background:** Mycophenolic acid (MPA) is an important immunosuppressive drug (ISD) prescribed to prevent graft rejection in the organ transplanted patients, however, its use is also associated with adverse side effects like sporadic gastrointestinal (GI) disturbances. Recently, we reported the MPA induced tight junctions (TJs) deregulation which involves MLCK/MLC-2 pathway. Here, we investigated the global histone acetylation as well as gene-specific chromatin signature of several genes associated with TJs regulation in Caco-2 cells after MPA treatment.

**Results**: The epigenetic analysis shows that MPA treatment increases the global histone acetylation levels as well as the enrichment for transcriptional active histone modification mark (H3K4me3) at promoter regions of *p38MAPK, ATF-2, MLCK*, and *MLC-2*. In contrast, the promoter region of *occludin* was enriched for transcriptional repressive histone modification mark (H3K27me3) after MPA treatment. In line with the chromatin status, MPA treatment increased the expression of *p38MAPK, ATF-2, MLCK*, and *MLC-2* both at transcriptional and translational level, while occludin expression was negatively influenced. Interestingly, the MPA induced gene expression changes and functional properties of Caco-2 cells could be blocked by the inhibition of p38MAPK using a chemical inhibitor (SB203580).

**Conclusions**: Collectively, our results highlight that MPA disrupts the structure of TJs via p38MAPK-dependent activation of MLCK/MLC-2 pathway that results in decreased integrity of Caco-2 monolayer. These results led us to suggest that p38MAPK-mediated lose integrity of epithelial monolayer could be the possible cause of GI disturbance (barrier dysfunction) in the intestine, leading to leaky style diarrhea observed in the organ-transplanted patients treated with MPA.

## Introduction

Mycophenolate mofetil (MMF) and enteric-coated mycophenolate-sodium (EC-MPS) are two commercially available formulations of immunosuppressive regimens that contain active agent mycophenolic acid (MPA; Bunnapradist et al., 2014; Xu et al., 2014). MPA inhibits the activity of inosine monophosphate dehydrogenase (IMPDH), a vital enzyme in the *de novo* synthesis of guanine nucleotide, thus preventing the synthesis of DNA and thereby inhibits growth and division of rapidly growing cells such as lymphocytes of the immune system (Watts, 1983). This property makes MPA as an effective immunosuppressive regime to suppress the immune system in order to prevent graft rejection in organ transplanted patients. Though MPA is vital to suppress the immune system to prevent graft rejection, its use is linked to the gastrointestinal (GI) disturbances in the transplanted patients (for details, see review articles Helderman and Goral, 2002; Malinowski et al., 2011). Several studies have shown that defect in the intestinal barrier function due to MMF or EC-MPS treatment results in increased permeability of intestinal mucosa (epithelial monolayer) for the solutes (Bunnapradist et al., 2014), develop leak-flux diarrhea in the rat model (Xu et al., 2014), and in renal and kidney transplanted patients (Watts, 1983; Helderman and Goral, 2002).

RETRACTED

Gastrointestinal disturbances in inflammatory bowel diseases (IBD) like Crohn's disease and ulcerative colitis, and in graft vs. host disease are mainly characterized by epithelial monolayer barrier defects which contribute to enhanced intestinal permeability (Clayburgh et al., 2004) and subsequent translocation of infectious agents and/or endotoxin from gut (Deitch, 2002; Magnotti and Deitch, 2005). Epithelial cells are connected with each other by four different types of junctions called desmosomes, gap-, adheren-, and, tight- junctions (TJs; Costa et al., 2013; Hong et al., 2013; Siljamäki et al., 2014). TJs are complex structure of ~35 different proteins including integral membrane proteins (claudins, occludin, junctional adhesion molecules “JAMs”) and peripheral membrane proteins [Zonula Occludens (ZO) such as ZO-1, ZO-2, and ZO-3; Tsukita et al., 2001; Schneeberger and Lynch, 2004]. TJs assist to seal the paracellular space between the adjacent cells, and is particularly involved in regulating barrier and fence functions (Shen et al., 2011). In “barrier function,” TJs regulate the passage of ions, water, and various molecules through paracellular pathways. Thus, aberrant barrier function can cause edema, jaundice, diarrhea, and blood-borne metastasis, however, the cell polarity is maintained by forming a fence to prevent intermixing of molecules between apical and lateral membrane. It is interesting to note that the altered fence function is involved in cancer progression in terms of loss of cell polarity (Sawada, 2013).

RETRACTED

In GI tract, TJs opening is considered as a key limiting factor of mucosal paracellular movement of nutrients and solutes. Growing evidences have indicated that TJs opening is modulated by the phosphorylation of myosin light chain 2 (MLC2), which principally depends upon the activation of MLC kinase (MLCK). The MLCK itself is however triggered by different types of stimuli such as IFN-gamma, TNF-alpha, and LIGHT (Lymphotoxin-like inducible protein that competes with glycoprotein D for herpes virus entry on T cells). This stimulation results in contraction of cytoplasmic actin filaments and redistribution of TJs anchoring protein, ZO-1 and structural protein, occludin in IBD (Crohn's disease, ulcerative disease), leaky flux diarrhea, and cholera (watery diarrhea; Zolotarevsky et al., 2002; Utech et al., 2005; Schwarz et al., 2007; Marchiando et al., 2010; Qasim et al., 2014). Recently, it has been shown that proinflammatory cytokine (IL-1β) induces TJs permeability in both *in vitro* and *in vivo* models through *p38MAPK/ATF-2*-dependent regulation of *MLCK* activity (Al-Sadi et al., 2013). p38MAPK is activated by various cellular stress agents (i.e., UV irradiation, heat shock, osmotic stress, lipopolysaccharide, cytokines; Mittelstadt et al., 2005; Keren et al., 2006) and is known to play a vital role in apoptosis, cytokines production, transcriptional regulation, and cytoskeletal reorganization (Kelkar et al., 2005; Lee and Dominguez, 2005; Baan et al., 2006). Previously, we reported that MPA alters TJs assembly in Caco-2 monolayer, similar to GI tract, via MLCK/MLC-2 pathway (Qasim et al., 2014).

The aim of the present study was to investigate whether MPA treatment leads to increased TJs permeability via p38MAPK dependent MLCK/MLC-2 pathway in MPA-treated Caco-2 cells monolayer.

## Materials and methods

### Experimental design

We used Caco-2 cells as a model cell line to investigate the MPA-mediated TJs modulation via p38MAPK dependent MLCK/MLC-2 pathway. Toward this, we established three groups: (1). MPA-treated group, (2). SB+MPA-treated group, and (3). DMSO (control)-treated group of differentiated and polarized Caco-2 cells monolayers. Each group was treated with MPA or SB+MPA or DMSO for 72 h. Different molecular analyses (epigenetic, mRNA expression, protein expression, and phosphorylation status) and functional analyses (TEER and FITC-Dextran dye flux) were performed to explore the role of p38MAPK-dependent MLCK/MLC-2 pathway in maintaining epithelial monolayer integrity following MPA treatment.

### Chemicals/reagents

Cell culture media Dulbecco's Modified Eagle's medium (DMEM), fetal calf serum (FCS), phosphate buffer saline (PBS), penicillin and streptomycin were purchased from PAA Laboratories, Pasching, Austria. Fluorescein isothiocyanate-conjugated dextran (FITC-dextran), 4 kDa (FD4), Trypsin, MPA, and DMSO were purchased from Sigma-Aldrich, Steiheim, Germany. Protease and phosphatase inhibitor cocktails were purchased from Roche, Mannheim, Germany. Bromophenol blue was obtained from Carl Roth, Karlsruhe, Germany. Sodium dodecyl sulfate (SDS) was obtained from Serva, Heidelberg, Germany. Glycerin, potassium ferricynaide, and sodium thiosulfate were purchased from Merck, Darmstadt, Germany. Formic acid was purchased from BASF, Ludwigshafen, Germany. Magnesium chloride (MgCl_2_), M-MLV RT enzyme, and 5X PCR buffer were from Invitrogen, Karlsruhe, Germany. Deoxynucleotide triphosphates (dNTPs) were from Roche, Mannheim, Germany and PCR primers were synthesized by Eurofins, Ebersberg, Germany. Ribonuclease (RNAase) inhibitor was obtained from Promega, Mannheim, Germany. The cell lysis buffer (10X) was obtained from Cell Signaling Technology, Danvers, MA, USA. All other chemicals used in this work were from the highest available purity from commercial sources unless otherwise stated.

RETRACTED

### Primer design

Promoter sequences were retrieved for each gene using Transcriptional Regulatory Element Database (TRED). Primer3 (v. 0.4.0) was used to design primers against promoter region and their specificity was checked by Human BLAT Search.

### Cell culture

All experiments were performed with human colon carcinoma (Caco-2) cells (Passages No. 15-25). Caco-2 cells were purchased from DSMZ (German collection of microorganisms and cell culture, Braunschweig, Germany) and grown in DMEM medium supplemented with 10% FBS, 1% Penicillin/Streptomycin, 1% non-essential amino acids. Confluent monolayers were obtained within 3–5 days after cell seeding (2 × 10^5^ cells/cm^2^) and grown further for 13 days (d) post-confluency. Medium was changed every other day after formation of confluent monolayer. Three groups were established i.e., MPA-treated, SB203580 (SB)+MPA-treated, and DMSO treated (control group). Cells were washed with PBS prior to the 72 h exposure with either MPA (10 μM) or DMSO. In case of SB (10 μM) treatment, cells were incubated with SB 1 h prior to the addition of MPA.

### Caco-2 monolayer integrity assays

#### Determination of trans-epithelial electrical resistance (TEER)

The intactness of paracellular pathways that control small molecules movement across Caco-2 monolayer was examined by TEER as previously described (Feldman et al., 2007; Qasim et al., 2014). Briefly, Caco-2 cells were seeded on polyester transwell inserts (6.5 mm diameter, 0.33 cm^2^ growth surface area, 0.4 μm pore size; Corning Costar corporation, USA) at a density of 2 × 10^5^ cells/well. Stable TEER of confluent monolayer was achieved at days 13–15 after seeding. Caco-2 plated filter having constant TEER (≥400 Ω.cm^2^) were included in experiments. Post-confluence monolayers having stable TEER were treated with MPA or SB plus MPA or DMSO (control) for 72 h. TEER was measured at 0, 12, 24, 48, and 72 h time period using an epithelial voltammeter (EVOM2, World Precision Instruments) with a STX2 electrode (World Precision Instruments, FL, USA). The TEER-values were normalized against background resistance of a blank insert that contained only medium. TEER was measured as ohms × cm^2^ (Ω.cm^2^) using the following formula: Resistance (TEER) = [*RC – RE*] × *A*, where *RC* is resistance of the cells (Ω); *RE* is resistance of the blank (Ω); *A* is surface area of the membrane insert (cm^2^). The results were expressed as the change in TEER with respect to time-matched controls [ΔTEER (Ω.cm^2^)]. TEER-values were calculated in three independent biological replicates each performed in duplicates.

RETRACTED

#### Fitc-dextran assay (FD4)

After 72 h of incubation with MPA or SB plus MPA or DMSO, permeability of Caco-2 monolayers was assessed using a previously reported dye fluxes method (Schlegel et al., 2011; Qasim et al., 2014). Briefly, Caco-2 cells were grown into monolayers and treated as described above. Following MPA treatment, monolayers were rinsed carefully with Hank's balanced salt solution (HBSS). To measure paracellular permeability (apical to basolateral fluxes), HBSS containing 1 mg/mL FD4 solution was added to the apical side for 2 h. Permeability marker flux was assessed by taking 100 μL from the basolateral chamber after 0, 20, 40, 60, 80, 100, and 120 min. Fluorescent signal was measured using a Lambda fluoro 320 fluorescence plate reader (MWG Biotech, Ebersberg, Germany) using 492 nm excitation and 520 nm emission filters. Standard curve, generated by serial dilution of FD4, was used to determine the FD4 flux concentrations across the monolayer. The flux concentration, which represents the permeability of monolayer, in the basolateral chamber was calculated by the following formula “Papp = [(ΔC_A_/Δt) V_A_]/AC_L_.” Where Papp is the apparent permeability (cm/s), ΔC_A_ is the change of FD4 concentration, A is the surface area of the membrane (cm^2^), Δt is the change of time, V_A_ is the volume of the abluminal medium, and C_L_ is the initial concentration in the luminal chamber. FD4-values were calculated in three consecutive experiments, each performed in duplicates.

### RNA expression analysis

Cells were grown for 13 d post-confluence and treated for 72 h in six-well plates as described above. Trizol (Trizol reagent; Invitrogen, USA) was used to extract total cellular RNAs from Caco-2 cell monolayers (MPA-treated or SB plus MPA-treated or DMSO-treated) according to the manufacturer's instructions. Briefly, Caco-2 monolayers were rinsed with ice-cold PBS and harvested by scraping with a rubber policeman into Trizol reagent, homogenized by inverting the tube twice, and RNA was extracted using chloroform/isopropanol precipitation. The precipitated RNA was air dried, dissolved in sterile water and stored at –80°C until analysis. RNA was quantified using a NanoDrop 2000C (PeqLab, Thermo Scientific).

RETRACTED

Reverse transcription reaction was performed using 1 μg of total RNA in a 30 μL reaction mixture containing 1X RT-PCR buffer [10 mmol/L Tris–HCl (pH 8.3), 15 mmol/L KCl, 0.6 mmol/L MgCl 2], 0.5 μmol/L of each dNTP, 1 U/μL RNase inhibitor and 13.3 U/μL M-MLV RT enzyme. The RT reactions were performed in a thermocycler (Biometra, Goettingen, Germany) at 65°C for 5 min, 37°C for 52 min, and then inactivated by heating at 70°C for 15 min. cDNA was stored at −80°C until use. Online Primer 3 software was used to design primers for the amplification of target genes by real time PCR (Rozen and Skaletsky, 2000; For primers used in this study see Table 1).

**Table 1:** **Promotor assay and mRNA expression primer list**.

**Name**	**Chromosomal location**	**Direction**	**Promoter assay primers**		**Expression primers**	
			**Sequences**	**Product size (bps)**	**Sequences**	**Product size (bps)**
p38MAPK	6	Forward	TTTGACTCTTTCCCCGACAC	187	CCAGCTTCAGCAGATTATGC	246
		Reverse	AACTGGAGACCAAAGGCAGA		TGGTACTGAGCAAAGTAGGCA	
ATF-2	2	Forward	CCTCAGCATACTGGTGCATT	159	GGCTTCTCCAGCTCACACA	326
		Reverse	TGGATGTGCTGACCGAACTA		TGTTTCAGCTGTGCCACTTC	
MLCK	3	Forward	TCTGCTGCAGTTCAGAGCAA	150	GATGATGCTCCAGCCAGT	177
		Reverse	AGGAGGAATGGTCAACAGCA		GTCCTCAGGGAACTGGATGA	
MLC-2	12	Forward	TCCACCTCCATCTTCTTTGC	168	AGAGACACCTTTGCTGCCCTT	188
		Reverse	GCCTTTGCCTTCCTTACACA		CCTTTGCCTTCAGGGTCAAAC	
Occludin	5	Forward	TGGATGGCAACTAACACCTACA	142	TGGGACAGAGGCTATGGAAC	287
		Reverse	AACGAAAGACTCCTGGGAAAAT		ATGCCCAGGATAGCACTCAC	
ZO-1	15	Forward	GCACATCAGCACGATTTCTG	166	TGAGGCAGCTCACATAATGC	224
		Reverse	AAACAGTGGGCAAACAGACC		GGTCTCTGCTGGCTTGTTTC	
GAPDH	12	Forward	TGAGCAGTCCGGTGTCACTA	152	ACCCAGAAGACTGTGGATGG	201
		Reverse	ACGACTGAGATGGGGAATTG		TTCTAGACGGCAGGTCAGGT	

Light Cycler instrument (Roche, Manheim, Germany) was used to amplify cDNA in a 20 μL reaction mixture containing 1 μL of cDNA solution, 2 μL of 10X PCR buffer (Invitrogen, Darmstadt, Germany), 2 μL SYBR green, 1 μL DMSO, 0.25 μL of each primer, 2.0 mmol/L MgCl_2_, 0.2 mmol/L of each dNTP, and 0.15 U/μL PAN Script DNA polymerase (PAN Biotech, Aidenbach, Germany). The following conditions were set to amplify cDNA; [(denaturation: 95°C for 5 min, one cycle); (40 cycles, denaturation: 95°C for 30 s, (annealing: *p38MAPK* (56°C), *ATF-2* (57°C), *MLCK* (56°C), *MLC-2* (57°C), *occludin* (57°C), *ZO-1* (57°C), and *GAPDH* (60°C) for 30 s), extension (72°C) for 30 s)].

RETRACTED

PCR data was normalized using internal control gene (GAPDH) and comparative Ct method (2^−ΔΔCt^; Schmittgen and Livak, 2008) was used to calculate the alteration of relative mRNA expression as a fold change between MPA treated and control cells. Amplified PCR product specificity was further confirmed by running on 1.5% agarose gel electrophoresis. Three separate experiments were performed with each one in triplicates.

### Dot blot

Dot blot assay was performed as described previously (Bölin et al., 1995) with little modification. Briefly, Caco-2 cells were cultured into differentiated and polarized monolayers and treated with the therapeutic concentration of MPA or DMSO for 72 h. Total cell lysate was prepared by 1X lysis buffer (Cell Signaling) at 0, 1, 12, 24, 48, 72 h. Proteins were quantified by Bio-Rad protein assay kit according to the manufacturer's guidelines. One centimeter square (cm^2^) grid was drawn by pencil on nitrocellulose membrane. Two microliters (protein concentration 10 μg/μl) of each sample was slowly spotted into the center of grid using narrow-mouth pipette tips. Sample spotted membranes were dried at RT. Non-specific binding sites were blocked by soaking sample spotted membrane in 5% BSA in TBST for 1 h at RT on a plate shaker at low speed. Each membrane was incubated with primary antibody (05 μg/ml rabbit anti-H3K9ac—Abcam or 1:20,000 rabbit anti-H4K8ac—Diagenode) dissolved in 5% BSA/TBST for 2 h at RT on a plate shaker at low speed. Following incubation with primary antibodies, each membrane was washed three times for 5 min and then incubated with secondary antibodies conjugated with HRP for 1 h at RT on a plate shaker at low speed. Then the membrane was washed three times and incubated with ECL reagents for 2 min, covered with saran-wrap and exposed to X-ray film in the dark room for different time, and proceeded for autoradiography using Konica SRX-101A (Konica Minolta).

### Western blot

Caco-2 cells were cultured into differentiated and polarized monolayers and treated as described above and were rinsed and collected with ice-cold PBS. Cells were lysed with lysis buffer-CS (50 mM Tris/HCl, pH 7.4, 1.0% Triton X-100, 5 mM EGTA, 10 mM sodium fluoride, 2 μg/mL leupeptin, 10 μg/mL aprotinin, 10 μg/mL bestatin, 10 μg/mL pepstatin A, 1 mM vanadate, and 1 mM PMSF). Total proteins (cleared supernatant) were separated by centrifugation from the cell lysate. Protein concentrations were measured using Bio-Rad protein assay kit (Bio-Rad Laboratories) according to the manufacturer's guidelines. Total protein contents were separated by 12.5% SDS-PAGE and blotted onto PVDF membrane (0.45 μm pore size, Immobilon, Millipore, MA, USA) using Trans-Blot SD cell system (Bio-rad, Munich, Germany) for 30 min at 15 V in a blotting buffer [192 mmol/L glycine, 20% methanol, and 25 mmol/L Tris (pH 8.3)]. To prevent nonspecific binding sites, each membrane was blocked with 5% milk (w/v) in TBS-T buffer [50 mmol/L Tris–HCl (pH 7.5), 200 mmol/L NaCl, 0.05% Tween 20] for 1 h at room temperature. Blocked membranes were washed twice in TBS-T for 5 min, then incubated with following antibodies: 1:10,000 dilution of mouse monoclonal anti-MLCK antibody (Sigma, Mannheim, Germany), 1:500 dilution of a mouse monoclonal anti-MLC-2 antibody (Sigma, Mannheim, Germany), 1:1000 rabbit anti-phospho MLC-2 antibody (Cell Signaling, Beverly, USA), 1 μg/mL rabbit anti-ZO-1, 0.5 μg/mL mouse anti-occludin (Zymed, CA, USA), 1:500 dilution of rabbit anti-H3K9ac (abcam), 1:250 dilution of H4K8ac (diagenode), or 1:5000 anti-β actin (Sigma, Mannheim, Germany) in 5% BSA in TBS-T for overnight at 4°C. Following overnight incubation with primary antibodies, membranes were washed with TBS-T buffer and again incubated with appropriate HRP-conjugated secondary antibodies (Bio-Rad, Munich, Germany), then washed with PBS and arranged for enhanced chemiluminescence detection (GE, Buckinghamshire, UK) according to the manufacturer's recommendation. The chemiluminescence signal was captured by hyperfilm-ECL (GE, Buckinghamshire, UK) and visualized using Konica SRX-101A (Konica Minolta). The densities of the specified protein bands between MPA-treated, SB plus MPA and control samples were quantified using ImageJ software (v 1.48, NIH, USA).

RETRACTED

### Chromatin immunoprecipitation (ChIP)

Caco-2 cells were cultured and treated as earlier described in “cell culture.” For ChIP analysis, cells were fixed with formaldehyde at a final concentration of 1.0% for 30 min at room temperature to cross-link DNA binding proteins and DNA (Boyd et al., 2009). Cells were harvested with ice cold PBS and counted by Advia 120 (Siemens) and equal number of cells were lysed according to the manufacturer's instructions (Red ChIP Kit™, Diagenode). Cross-linked chromatin was sheared into fragments of 100–1000 bps using Branson Sonifier 250 for 3 min using cycles of 30 s sonication and 1 min on ice. One-tenth of the sample was set aside as an input control, and the rest was pre-cleared with protein A magnetic beads for 30 min at 4°C with agitation. Pre-cleaned chromatin was then precipitated with active histone mark antibody (H3K4me3, Abcam, ab8580), as well as with repressive histone mark antibody (H3K27me3, Millipore, 07-449), and normal IgG (One Day ChIP Kit™, Diagenode) from both treated and untreated cells. The Chromatin-antibodies-magnetic beads complexes were washed with 1X ChIP washing buffer (One Day ChIP Kit™, Diagenode). Proteinase K was used to degrade the DNA associated proteins and DNA was isolated by DNA slurry (One Day ChIP Kit™, Diagenode) and quantified by NanoDrop (NanoDrop 2000C, peqlab, Thermo Scientific). ChIP-precipitated genomic DNA was amplified using real time PCR (Roche, Manheim, Germany) in 20 μL SYBR green based reaction (For promoter based primers see details in Table 1). PCR amplification was done under the following conditions; [(denaturation: 95°C for 2 min, one cycle); (40 cycles, denaturation: 95°C for 30 s, (annealing: p38MAPK (60°C), ATF-2 (55°C), MLCK (62°C), MLC-2 (62°C), occludin (54°C), ZO-1 (55°C), and GAPDH (59°C) for 30 s), extension (72°C) for 30 s)].

### Data analysis

Ct-values from real time PCR were analyzed by “input percent method” (Lin et al., 2012). Briefly, raw Ct-value of the diluted input (1%) was adjusted to 100% by subtracting the dilution factor of 100 or 6.644 cycles (i.e., log2 of 100). Sample raw Ct-values (ΔCt) were normalized by subtracting adjusted Input (Ct Input –6.644) Ct-value. And finally the “Input percent” value for each sample was calculated using the following formula. Input % = 100 ^*^ 2ˆ(adjusted input – Ct IP). The “Input percent” value represents the enrichment of H3K4me3 and/or H3K27me3 at the promoter region of genes studied. Dissociation curve analysis was performed to confirm the specificity of each PCR product. GAPDH was used as an internal control gene.

### Statistics

Statistical program GraphPad (GraphPad, San Diego, CA) was used to perform statistical analysis. Data was analyzed by analysis of variance (ANOVA) and comparisons between control and MPA treatment were made using the Bonferroni posttest. Alternatively, statistical significance between control and treatment group were calculated using student's *t*-test. Results were expressed as mean ± standard error of the mean (SEM). Probability of 0.05 or less was deemed statistically significant (^*^P < 0.05, ^**^P < 0.01, ^***^P < 0.001).

## Results

### MPA increases global histone (H3K9 and H4K8) acetylation in Caco-2 cells

Acetylation of histone proteins plays an important role in the unfolding of chromatin and initiation of transcription. Recently it was reported that MPA treatment increases the histone H3/H4 global acetylation levels in CD4^+^ T cells from systemic lupus erythematosus patients (Yang et al., 2015). In order to study whether MPA treatment leads to similar epigenetic changes also in epithelial monolayer, Caco-2 cells monolayers were treated with MPA for various time points and analyzed for global histone acetylation levels using dot- and Western -blot analysis. The dot blot results show that MPA treatment increases global acetylation of H3K9 and H4K8 in Caco-2 cells after 72 h (Figure 1A). Western blot analysis further confirmed that MPA significantly increases the acetylation of H3K9 and H4K8 after 72 h (Figures 1B–D). These results indicate that MPA treatment significantly alters the epigenetic status of Caco-2 cells.

RETRACTED

**Figure 1:** **MPA treatment increases global histone acetylation in Caco-2 cells**. **(A)** Dot-blot analysis; Caco-2 cells were cultured in six-well plates and post confluence monolayers were treated either with 10 μM MPA or DMSO for indicated time points. Total proteins were extracted and a volume of 2 μl from each time point was spotted on nitrocellulose membrane, dried and then probed with anti-H3K9ac and anti-H4K8ac antibodies. **(B)** Western blot analysis; Total cell proteins were resolved on 12.5% SDS-PAGE gels and, immunoblotted using anti-H3K9ac and anti-H4K8ac specific antibodies. β-actin was used as a loading control. **(C,D)** Bar graphs representing the densitometric analysis of three independent experiments from Western blot **(B)** using the Lab image software. Differences between two groups were analyzed by the two-tailed Student's *t*-test and of more than two groups by One-way ANOVA with Bonferroni posttest (*n* = 3) and the values were expressed as means ± SEM. Asterisk indicates the significance (^***^P < 0.001) when compared to control cells. ns, non-significant.

### MPA treatment activates MLCK and MLC-2 while inactivates occludin at epigenetic level in Caco-2 cells

We and other investigators have reported the involvement of MLCK pathway in the regulation of TJs barrier function (Cunningham and Turner, 2012; Qasim et al., 2014). In light of the global increase in histone acetylation levels after MPA treatment, we assessed the epigenetic status at the promoter region of *MLCK, MLC-2, occludin*, and *ZO-1* genes, by ChIP assay in MPA treated or untreated Caco-2 monolayer cells. Our ChIP data showed that the transcription permissive histone modification mark (H3K4me3) was increased significantly at the promoter region of *MLCK* and *MLC-2* genes, respectively (Figures 2A,B). Concomitantly, transcription repressive mark (H3K27me3) was decreased significantly at the promoter region of *MLCK* and *MLC-2* genes, respectively, as compared to controls (Figures 2A,B). While promoter of *occludin* lost H3K4me3 mark and gained H3K27me3 mark in the MPA treated Caco-2 cells as compared to control cells, indicating the transcriptional silencing of *occludin* after MPA treatment (Figure 2C). However, the promoter region of *ZO-1* showed no significant changes in H3K4me3 and H3K27me3 levels between MPA-treated cells and control (Figure 2D).

RETRACTED

**Figure 2:** **MPA causes epigenetic alteration of *MLCK/MLC-2* pathway and tight junction genes (*occludin*)**. **(A–D)** Caco-2 cells were grown for 13 days post-confluence to form differentiated monolayers and then treated for 72 h with MPA or DMSO. ChIP was performed using anti-H3K4me3 (activation mark) or anti-H3K27me3 (repression mark), followed by real time PCR using promoter-specific primers of the target genes (*MLCK, MLC-2, Occludin*, and *ZO-1*). Levels of H3K4me3 or H3K27me3 was measured as %age input in the MPA treated cells as compared to the untreated cells. **(E,F)** Western blot analyses of MLCK, MLC-2, occludin, and ZO-1 after MPA treatment. Whole cell protein lysates were resolved on SDS-PAGE gels and immunoblotted using of anti-MLCK, anti-MLC-2, anti-occludin, and anti-ZO-1 specific antibodies. β-actin was used as a loading control for an equal amount of protein. Densitometric analysis was done using the Lab image software on three independent experiments. Differences between two groups were analyzed by the two-tailed Student's *t*-test and of more than two groups by One-way ANOVA with Bonferroni posttest. **(G)** DMSO treated Caco-2 monolayer cells. The values were expressed as means ± SEM. Asterisk indicates the significance (^**^P < 0.01, ^***^P < 0.001) when compared to control cells. (*n* = 3). ns, non-significant.

To confirm the influence of MPA on the epigenetic activation of *MLCK* and *MLC-2* genes, transcriptional and translational expression was analyzed using quantitative PCR and immunoblotting, respectively. In line with the earlier reports (Qasim et al., 2011, 2014), MPA treatment significantly increased the expression of MLCK and MLC-2 both at transcriptional and protein level (Figures 2E–G). Further we analyzed the expression of occludin to confirm the epigenetic data at mRNA and protein level and found significant decrease at protein and mRNA expression (Figures 2E–G). In contrast, we did not observe any significant difference in ZO-1 RNA or proteins expression in MPA-treated Caco-2 cells as compared to control cells (Figures 2E–G). Collectively, the gene expression data correlate well with the gene-specific epigenetic changes induced by MPA treatment in Caco-2 monolayer cells.

RETRACTED

### MPA treatment activates p38MAPK and ATF-2 at epigenetic level in Caco-2 cells

Recently it was reported that p38MAPK increases TJs permeability in IL-1β treated Caco-2 through activation of MLCK pathway (Al-Sadi et al., 2013). In this study we aimed to extend our previous knowledge and explored whether p38MAPK acts upstream of MLCK/MLC-2 pathway in MPA-treated Caco-2 cells. Toward this end, firstly, we assessed the epigenetic status of *p38MAPK* and *ATF-2* genes at their promoter regions by ChIP assay in MPA treated or untreated Caco-2 monolayer cells. Our ChIP results showed that the activation histone modification mark (H3K4me3) was increased significantly at the promoter region of *p38MAPK* and *ATF-2* genes, respectively, in MPA treated cells (Figures 3A,B). Concomitantly, repression mark (H3K27me3) was decreased significantly at the promoter region of *p38MAPK* and *ATF-2* genes, respectively, as compared to controls (Figures 3A,B). The transcriptionally active epigenetic state of *p38MAPK* and *ATF-2* was confirmed by the mRNA expression analysis that showed significant increase in *p38MAPK* and *ATF-2* expression after MPA (Figure 3C).

**Figure 3:** **p38MAPK regulates MLCK/MLC-2 pathway and its inhibition partially prevents MPA-induced TJs dysfunction**. **(A,B)** Epigenetic status at the promoter regions of *p38MAPK* and *ATF-2* genes MPA or DMSO treated Caco-2 monolayer cells. ChIP was performed with antibodies specific to the activation mark (H3K4me3) or repression mark (H3K27me3), followed by real time PCR analysis. Relative intensity of activation mark (H3K4me3) or repression mark (H3K27me3) were measured as %age input. **(C)** Bar graph showing the p38MAPK and ATF-2 mRNA expression. **(D–H)** Western blots and the corresponding densitometric data showing the effect of SB on the expression of MLCK/MLC-2 pathway and tight junction proteins (occludin and ZO-1). **(I,J)** Line graphs showing the transeplithelial electrical resistance (TEER) **(I)** and paracellular flux (FITC-dextran) **(J)** assay results obtained either in presence or absence of p38MAPK inhibitor. Error bar indicate means ± SEM. Asterisk indicates the significance (^*^P < 0.05, ^**^P < 0.01, ^***^P < 0.001) when compared to control cells. (*n* = 3). ns, non-significant.

### Inhibition of p38MAPK via SB counteracts the altered expression of MLCK, MLC-2, and occludin genes in MPA-treated Caco-2 cells

In order to test whether MPA indeed regulates p38MAPK-dependent expression of MLCK pathway and thereby the TJs defects, we performed the p38MAPK inhibition and studied its effect at the functional level. The chemical inhibitor SB203580 (SB), a representative of pyridinlimidazole, is a specific inhibitor of p38MAPK and is widely used in inhibitory studies to attenuate the activity of p38MAPK and its downstream signaling activities in various physiological processes (Kumar et al., 1999). Our results showed that p38MAPK inhibition in MPA treated Caco-2 cells prevented any significant change in expression of MLCK, MLC-2, phosphorylated MLC-2 (pMLC-2), and Occludin protein as compared to DMSO only treated cells (Figures 3D–G). While the expression of ZO1 was found unaltered by MPA or MPA+SB treated Caco-2 cells (Figure 3H).

RETRACTED

### p38MPAK inhibition partially reverses MPA-induced TJs dysfunction

The maintenance of normal protein levels of MLCK, MLC2, and occludin after p38MAPK inhibition prompted us to study the functional properties of Caco-2 monolayer in the presence of SB. The intactness of Caco-2 cells differentiated into polarized confluence monolayer can be measured quantitatively as TEER-value and the sum of the resistance indicates the integrity of the monolayer barrier maintained by TJs in the apical surface of the cells. Any damage to the intactness of monolayer results in reduced TEER-value. In accordance with the literature, exposure of Caco-2 monolayer to MPA significantly decreased TEER at 24 h after treatment, and the TEER was significantly further decreased by 72 h as compared to the control cells (Figure 3I). Similarly, FD4 permeability analysis (traditionally used to measure the movement of small molecules across the intestinal epithelium *in vivo*) following 72 h MPA treatment showed a time-dependent increase across (from the apical to the basolateral side) the Caco-2 monolayer, as expected (Figure 3J).

Interestingly, when MPA-treated Caco-2 cells monolayers were co-incubated with the inhibitor for p38MAPK, very significant preservation of TEER (~50%) was observed as compared to only MPA-treated Caco-2 cells (Figures 3I,J). Similarly, 50% reduction in the FD4 leak on the basolateral side of the Caco-2 cell monolayer was measured as compared to only MPA-treated monolayer (Figure 3J). Collectively, these results confirm that the Caco-2 monolayer paracellular permeability is significantly increased after MPA exposure and that can be antagonized by blocking the activity of p38MAPK pathway.

### Inhibition of p38MAPK through SB demolishes increased promoter activity of downstream targets of p38MPAK in MPA-treated Caco-2 cells

Next, we analyzed whether the protein expression changes seen after the inhibition of p38MAPK are due to the epigenetic remodeling at the promoter regions of these genes or are due to protein stability. In accordance with the expression data of downstream targets of p38MAPK, the epigenetic signature at the promoter regions of *MLCK, MLC-2*, and *Occludin*, but not *ZO1*, was restored to the epigenetic status seen in control cells (Figures 4A–D) by SB use. Similarly, by use of SB, the promoter region of *ATF2*, but not *p38MAPK*, showed the normal chromatin signature seen in control cells (Figures 4E,F). These results were further confirmed by mRNA expression analysis, which showed that pretreatment with SB restored the MPA induced gene expression changes in Caco-2 cells while it had no significant inhibitory effects on mRNA expression of the *p38MAPK* gene (Figures 5A–C).

RETRACTED

**Figure 4:** **Inhibition of p38MAPK counteracts MPA-mediated epigenetic remodeling**. Effect of SB203580 on promoter activity of p38MAPK mediated MLCK/MLC-2 pathways and TJs genes in MPA-treated Caco-2 Cells. **(A–F)** Bar graphs showing the epigenetic status at the promoter regions of *MLCK, MLC-2, occludin, ZO-1, p38MAPK*, and *ATF-2* genes in either presence or absence of p38MAPK inhibitor. The ChIP-qPCR data was expressed as means ± SEM. Asterisk indicates the significance (^**^P < 0.01, ^***^P < 0.001) when compared to control cells. Differences between two groups were analyzed by the two-tailed Student's *t*-test and of more than two groups by One-way ANOVA with Bonferroni posttest. ns, non-significant.

**Figure 5:** **p38MAPK inhibition preserves normal MLCK/MLC-2 gene expression in Caco2 cells treated with MPA**. Bar graphs showing the mRNA expression levels of *MLCK* and *MLC-2* **(A)**, *occludin* and *ZO-1* **(B)**, and *p38MAPK* and *ATF-2* **(C)** in either presence or absence of p38MAPK inhibitor. Values are expressed as means ± SEM. Asterisk indicates the significance (^**^P < 0.01, ^***^P < 0.001) when compared to control cells. Differences between two groups were analyzed by the two-tailed Student's *t*-test and of more than two groups by One-way ANOVA with Bonferroni posttest. ns, non-significant.

## Discussion

Regulation of TJs barrier function, that controls paracellular movement, is a vital and complex process involving complicated intracellular signaling pathways and organization of TJs proteins leading to influence the passage of ions and solutes via paracellular movement across the epithelial monolayer (Anderson and Van Itallie, 1995; González-Mariscal et al., 2008). On the basis of initial morphological descriptions, TJs were characterized as a defined structure, both physiologically and morphologically (Farquhar and Palade, 1963). However, later it was accepted that TJs are a dynamically regulated structure (Pappenheimer, 1987; Taylor et al., 1998). The barrier function of epithelial monolayer depends upon the continuity of the monolayer and intact TJs (Anderson and Van Itallie, 1995, 2009; Hering et al., 2012). Intestinal barrier dysfunction through TJs disruption is characterized by increased paracellular permeability along with altered expression and organization of TJs proteins (Clayburgh et al., 2004; Prasad et al., 2005). Subsequently, other investigators and we have reported MLCK activation, which directly leads to the phosphorylation of MLC-2, as a common final pathway of acute TJs regulation in response to a broad range of physiological or pathophysiological stimuli (Turner, 2006, 2009; Qasim et al., 2014). Phosphorylation of MLC-2 through activated MLCK alone is sufficient to increase TJs permeability, which is associated with redistribution of ZO-1 and occludin (Al-Sadi et al., 2013). Previously, we have shown that therapeutic dose of MPA caused the increased permeability of Caco-2 monolayer, and this outcome is accompanied by increased activity of *MLCK/MLC-2 pathway* (Qasim et al., 2014). In this context, it is interesting to note that proinflammatory cytokine (IL-1β) induced increase in intestinal TJs permeability in both *in vitro* and *in vivo* models is mediated through *p38MAPK/ATF-2*-dependent regulation of *MLCK* activity (Al-Sadi et al., 2013). In this study, we wanted to extend our previous knowledge of TJs regulation via MLCK pathway in response to MPA. Our data highlight that MPA alters the chromatin structure leading to deregulated expression of genes implicated in TJs function. We identified that p38MAPK and ATF-2 pathway is activated in MPA treated Caco2 monolayer and this pathway was found regulate the MLCK/MLC-2 activity. Interestingly, pharmacological inhibition of p38MAPK counteracted the altered gene expression of MLCK/MLC-2 and thereby maintained the normal function of TJs. Chromatin structure is modulated by the well documented posttranslational modification of histone proteins (Strahl and Allis, 2000). More than 100 different types of posttranslational modifications that include; acetylation, methylation, phosphorylation, and ubiquitination can occur to the amino-terminal tails of histones, which form the nucleosomes of chromatin (Bernstein et al., 2007; Kouzarides, 2007). Majority of these modifications remain poorly understood, however, considerable progress has been made in the understanding of lysine acetylation and methylation of histones in recent years. Lysine acetylation is mostly correlated with nucleosome assembly, chromatin accessibility and transcriptional activity, whereas lysine methylation effects depend upon the modified residue (Bernstein et al., 2007). Acetylated H3K9 (Nishida et al., 2006) and H4K8 are well-known epigenetic markers that are present at the promoter regions of transcriptionally active genes (Gupta et al., 2013). Their levels are strongly correlated with the gene expression therefore referred as “transcription-linked” histone marks (Suzuki et al., 2008; Gupta et al., 2013). Our global histone acetylation analysis showed significant increase in acetylation at H3K9 and H4K8. This global chromatin change observed after MPA treatment is in agreement with a recent report showing that MPA treatment induces global H3/H4 acetylation in CD4(+)T cells to exert therapeutic effects in systemic lupus erythematosus patients (Yang et al., 2015). In this context, it is interesting to note that hydroxamic acid derivatives of MPA were shown to function as histone deacetylase (HDAC) inhibitors (Batovska et al., 2008). Owing to these evidences, it is interesting to speculate that MPA might exert its therapeutic effect on immune cells not only by blocking IMPDH, but also by acting as epigenetic modifier. And this epigenetic effect might also occur in non-immune cells such as epithelial cells leading to gene expression changes and unwanted phenotypic changes.

RETRACTED

Trimethylation of H3K4 is found at more than 90% of the RNA polymerase II binding regions (Barski et al., 2007) at the promoter region of protein coding genes and is linked to gene activation, whereas trimethylation of H3K27 is linked to repression of the gene (Barski et al., 2007; Guenther et al., 2007). Our ChIP-qPCR data showed significant enrichment of H3K4me3 at the promoter regions of MLCK and MLC-2 genes, enrichment of H3K27me3 at the promoter region of Occludin, while no change in H3K4me3 and H3K27me3 levels at ZO-1 promoter region after MPA treatment. The gene expression analyses at transcriptional and translational level further strengthened the epigenetic activation of *MLCK* and *MLC-2* genes and repression of *occludin* gene. Interestingly, Inhibition of p38MAPK with SB prevented the MPA mediated epigenetic changes as well as the gene expression pattern. Presence of SB together with MPA, significantly but not completely reduced the MPA induced TJs permeability, suggesting role for additional signaling pathways/proteins in TJs deregulation in MPA-treated Caco-2 cells. In view of current data, it would be interesting to check whether p38MAPK conditional knockout mice could alleviate or completely block the MPA-mediated TJs dysfunction. Therefore, a more detailed analysis of TJs proteins regulation as well as their regulating pathway(s) is necessary to understand the mechanism of leak flux diarrhea in *in vitro* model that is comparable to *in vivo* model of MPA therapy.

RETRACTED

## Conclusions

In summary, this study provides new insights and an essential understanding into the mechanisms of MPA-mediated decrease in intestinal epithelial barrier function. Our data pointed out epigenetic activation of *p38MAPK, ATF-2, MLCK*, and *MLC-2* genes whereas repression of *occludin* gene at promoter level (Figure 6). To the best of our knowledge, this is the first *in vitro* experimental study that provides direct evidence to indicate the role of chromatin remodeling in the p38MAPK-dependent MLCK pathway activation in response to MPA exposure. From these results, it can be hypothesized that comparable barrier function modulations may occur in the patients under MPA therapy leading to GI tract complication in some organ transplanted patients.

**Figure 6:** **Proposed mechanism of MPA-induced TJs assembly deregulation in Caco-2 cells monolayer**. Proinflammatory cytokines (as observed in IBD) directly or through p38MAPK activate the MLCK pathway which leads to the altered TJs proteins contents and composition in TJs assembly, resulting in compromised epithelial barrier function. This compromised barrier function contributes to leaky style diarrhea in IBD patients. Identification of altered chromatin structure at *p38MAPK, ATF-2, MLCK*, and *MLC-2* promoter regions after MPA treatment allow us to assume that MPA either directly or through unknown mediators activates the p38MAPK cascade. Activation of the p38MAPK-dependent MLCK/MLC-2 pathway consequently reorganizes F-actin base cytoskeleton, redistribute ZO-1 and occludin proteins of TJs assembly, resulting in increased permeability of Caco-2 monolayer.

## Author contributions

NK and AA conceived the study. NK, MQ, and DP performed and analyze the data. NK, DP, LB, and AA participated in interpretation and drafting the manuscript. DP and AA supervised the study. All authors read and approved the final manuscript.

### Conflict of interest statement

The authors declare that the research was conducted in the absence of any commercial or financial relationships that could be construed as a potential conflict of interest.

## Abbreviations

MPA: mycophenolic acid
p38MAPK: p38 mitogen activated protein kinase
ATF-2: activating transcription factor-2
MLCK: myosin light chain kinase
MLC-2: myosin light chain-2
TJs: tight junctions
ZO-1: Zonula Occludins
IL-1β: Interleukin-1 beta
TNF-α: Tumor necrosis factor-alpha
INF-γ: Interferon-γ.
